# NEAT1 enhances MPP^+^‐induced pyroptosis in a cell model of Parkinson's disease via targeting miR‐5047/YAF2 signaling

**DOI:** 10.1002/iid3.817

**Published:** 2023-06-23

**Authors:** Hong Shen, Hui Song, Songlin Wang, Daojing Su, Qiang Sun

**Affiliations:** ^1^ Department of Encephalopathy Second People's Hospital Suzhou City Jiangsu Province China; ^2^ Department of Neurology, TaiHe Hospital Hubei University of Medicine Shiyan City Hubei Province China; ^3^ Department of Orthopaedic Rehabilitation, TaiHe Hospital Hubei University of Medicine Shiyan City Hubei Province China

**Keywords:** inflammasomes, nuclear paraspeckle assembly transcript 1, Parkinson's disease, pyroptosis

## Abstract

**Purpose:**

Parkinson's disease (PD) is the second most frequent neurodegenerative disease. The aim of our study is to explore the role and the regulatory mechanism of long noncoding RNA (lncRNA) NEAT1 in MPP^+^‐induced pyroptosis in a cell model of PD.

**Materials and Methods:**

MPP^+^‐treated SH‐SY5Y cells were used as an in vitro model of dopaminergic neurons for PD. Expression levels of miR‐5047 and YAF2 mRNA were determined through qRT‐PCR. TUNEL staining was carried out to analyze neuronal apoptosis. Luciferase activity assay was accomplished to analyze the combination of miR‐5047 with NEAT1 or YAF2 3ʹ‐UTR region. Besides, concentrations of IL‐1β and IL‐18 in supernatant samples were analyzed by using ELISA assay. Expression level of proteins were examined through Western blot.

**Results:**

NEAT1 and YAF2 expression were increased, while miR‐5047 expression was declined in the SH‐SY5Y cells treated with MPP^+^. NEAT1 was a positively regulator to SH‐SY5Y cells pyroptosis induced by MPP^+^. In addition, YAF2 was a downstream target of miR‐5047. NEAT1 promoted YAF2 expression via inhibiting miR‐5047. Importantly, the promotion of NEAT1 to SH‐SY5Y cells pyroptosis induced by MPP^+^ was rescued by miR‐5047 mimic transfection or YAF2 downregulation.

**Conclusion:**

In conclusion, NEAT1 was increased in MPP^+^‐induced SH‐SY5Y cells, and it promoted MPP^+^‐induced pyroptosis through facilitating YAF2 expression by sponging miR‐5047.

## Graphical abstract

NEAT1 was increased in the SH‐SY5Y cells treated with MPP+, and it promoted the MPP+‐induced pyroptosis through facilitating YAF2 expression by sponging miR‐5047.

## 1 INTRODUCTION

Over the last few decades, central nervous system diseases have become a major cause of disability worldwide. Clinical common central nervous system diseases include Alzheimer's disease, metastatic brain tumor, stroke and Parkinson's disease (PD).^1^ PD is the second most frequent neurodegenerative disease and is characterized by the non‐motor symptoms like cognitive impairment and gastrointestinal dysfunction and the motor symptoms like bradykinesia, postural instability and resting tremor.^2^, ^3^, ^4^ Ageing, genetic, and environment risk factors or other pathogenic factors lead to loss of neuron in several brain areas, especially in the substantia nigra.^5^, ^6^ Mutations of *LRRK2*, *PRKN*, *PINK1*, *ATP13A2*, and *DJ‐1* are several known pathogenic genes for PD.^5^, ^7^ Currently, although a great advance in the technology used in drug discovery has been made, development of the drugs used in PD treatment remains challenging, which are due to the complex pathogenesis of the disease.

Numerous lines of evidence indicate that chronic neuroinflammation is one of the mainly hallmarks of PD, while whether inflammation increasing is a consequence or a cause of PD remains unclear.^8^, ^9^ Pyroptosis has been first introduced by Cookson and colleagues in 2001. Pyroptosis is mediated by caspase‐1 and accompanied by the release of a series cytokine, such as interleukin (IL) ‐1β and IL‐18.^10^ During pyroptosis, activation of caspase‐1 can be induced by inflammasome, such as NLR family pyrin domain‐containing (NLRP) 3 or NLRP1 inflammasome.^11^, ^12^ It was reported that NLRP3 inflammasome‐ or pyroptosis‐related proteins was highly expressed in the 1‐methyl‐4‐phenylpyridinium (MPP^+^)‐treated SH‐SY5Y cells, and pyroptosis was activated in above cells.^13^ Inhibition of NLRP3 inflammasome‐mediated pyroptosis in 1‐methyl‐4‐phenyl‐1,2,4,5‐tetrahydropyridine (MPTP)‐induced PD mice model or in MPP^+^‐treated PC12 cells could effectively attenuate neuron apoptosis.^14^ Currently, the inflammasome type studied in the pathogenesis of PD is mainly mediated by NLRP3, but there are few studies on the role of NLRP1 inflammasome in development of PD. Chen et al.^15^ demonstrated that expression of NLRP1 is decreased in anti‐inflammatory drugs‐treated α‐synuclein‐stimulated BV‐2 cells.

The thorough annotation of the human genome by the GENCODE and ENCODE projects indicated that many transcription products of the human DNA are long noncoding RNAs (lncRNAs), and more than 10,000 lncRNAs have been identified.^16^, ^17^ A number of lncRNA is known to be involved in regulation of PD. For instance, Simchovitz et al. provided a new lncRNA LINC‐PINT that is increased in the substantia nigra of PD patients and other PD models may play a neuroprotective role in PD.^18^ Among multiple lncRNAs, role of nuclear paraspeckle assembly transcript 1 (NEAT1) in PD is contradictory, that has attracted particular interest. In our previous study, the results demonstrated that NEAT1 is highly expressed in the SH‐SY5Y cells treated with MPP^+^, and that silencing of NEAT1 obviously attenuates neuronal apoptosis induced by MPP^+^.^19^ SH‐SY5Y cells have been widely used as a cell model of dopaminergic neurons for PD research.^20^, ^21^ In addition, some studies reported that NEAT1 induces the activation of inflammasome and its‐mediated pyroptosis in different diseases.^22^, ^23^ In this study, MPP^+^‐treated SH‐SY5Y cells were used as in vitro model of PD. We probed the functions and the regulatory mechanism of NEAT1 in SH‐SY5Y cells pyroptosis induced by MPP^+^, thus to investigate the role and action mechanism of NEAT1 in PD development. Our work proved a new evidence for the potential of NEAT1 in PD treatment.

## 2 MATERIALS AND METHODS

### 2.1 Cell culture and treatment

In the current study, MPP^+^‐treated SH‐SY5Y cells were used to mimic PD in vitro. SH‐SY5Y cells were obtained from the ATCC. MPP^+^ was got from the Sigma Company, and was utilized to induce PD cell model at the dosage of 100 μM for 24 h. The complete Dulbecco's Modified Eagle medium (DMEM) medium used in our study is composed of basal DMEM medium (Gibco), 10% fetal bovine serum (Gibco), as well as 1% penicillin/streptomycin (Gibco). Here, the treated and untreated SH‐SY5Y cells were cultured in complete DMEM medium. NEAT1 small interfering RNA (siRNA), siRNA negative control, miR‐5047 mimics, mimics negative control, miR‐5047 inhibitor, inhibitor negative control, and YY1‐associated factor 2 (YAF2) siRNA were synthesized by GenScript Company. All above gene segments, NEAT1 overexpression plasmid, as well as empty plasmid were transfected into SH‐SY5Y cells using Lipofectamine 3000 reagent (Invitrogen).

### 2.2 Detection of proteins expression

Expression levels of pro‐caspase‐1, cleaved caspase‐1, YAF2, NLRP1 and adaptor apoptosis‐associated speck‐like (ASC) were determined using Western blot. Collected SH‐SY5Y cells were washed with 0.01 M PBS solution for twice. Then, the cells were broken using RIPA lysis solution (Solarbio) for protein extraction. Next, 20 μg of proteins for each group were separated on 12% SDS‐PAGE gels for 2.5 h, and were transferred into polyvinylidene fluoride membranes. After that, membranes were blocked with 5% fresh nonfat milk for 1 h followed by incubation with primary antibodies overnight at 4°C. The anti‐pro‐caspase‐1, anti‐ASC, anti‐NLRP1, anti‐ anti‐cleaved caspase‐1, and anti‐β‐actin (internal reference) antibodies were purchased from Abcam. All primary antibodies were diluted at a ratio of 1:2000 when used. Next day, membranes were maintained with secondary antibodies for 1 h at room temperature. Finally, an ECL kit was utilized to analyze protein bands.

### 2.3 Detection of NEAT1, miR‐5047, and YAF2 mRNA expression levels

Expression levels of NEAT1, miR‐5047, and YAF2 mRNA were measured using qRT‐PCR assay. SH‐SY5Y cells were collected, and were washed with PBS for twice. Then, total RNA was isolated using TRIzol reagent (Invitrogen), and was reversed transcribed into complementary DNA usage the First‐Strand Synthesis Kit (Invitrogen). Next step, qPCR experiments were accomplished using SYBR Green PCR Master Mix Kit (Invitrogen). All steps were carried out strictly according to the instructions. In this study, expression of NEAT1 and YAF2 mRNA normalized to *GAPDH*. U6 served as the internal reference for miR‐5047. Expression levels of NEAT1, miR‐5047, and YAF2 mRNA were calculated through −2^ΔΔ*C*^t method.

### 2.4 Determination of the apoptotic rate in SH‐SY5Y cells

Apoptotic rate of SH‐SY5Y cells was measured using TUNEL staining. SH‐SY5Y cells at a density of 5 × 10^4^ cells/well were inoculated into 24‐well plates, and were treated with MPP^+^ or transfected with gene segments for 24 h. After that, cells were fixed with 4% formaldehyde fixative buffer (Solarbio) for 1 h, and were washed with PBS solution. After incubation with 3% H_2_O_2_ solution for 15 min, the treated and untreated SH‐SY5Y cells were maintained with 0.1% Triton X‐100 in PBS solution for 10 min. Subsequently, apoptotic cells were marked by TUNEL solution (Solarbio) in accordance with the instruction. After incubation with DAPI solution in the dark for 5 min to mark nucleuses, the number of apoptotic cells (TUNEL‐positive cells) were counted using Image J software.

### 2.5 Detection of the interaction of miR‐5047 with NEAT1 or YAF2 3ʹ‐UTR

Dual‐luciferase activity assay was fulfilled to determine the combination of NEAT1 and miR‐5047, and the combination of miR‐5047 and YAF2 3ʹ‐UTR. Here, the wild‐type (WT) and the altered gene sequences of NEAT1 or YAF2 3ʹ‐UTR containing the binding sites with miR‐5047 were subcloned into luciferase reporter plasmid. The recombinant plasmids of NEAT1‐WT, NEAT1‐ altered, YAF2 3ʹ‐UTR‐WT, and YAF2 3ʹ‐UTR‐altered were transfected with miR‐5047 mimics or mimics negative control into 293T cells. Luciferase activity was determined by using Dual‐Luciferase Reporter Assay System (Promega).

### 2.6 Detection of the IL‐1β and IL‐18 levels in supernatant

Concentrations of IL‐1β and IL‐18 in supernatant of SH‐SY5Y cells were measured through ELISA assay according to the protocols of human IL‐1β ELISA kit and human IL‐18 ELISA kit (R&D Systems).

### 2.7 Statistical analysis

Results were analyzed by using the SPSS 20.0 software (IBM), and images were marked by utilizing the GraphPad Prism 6.0 software. Data were presented as mean ± SD of three independent experiments. Student's *t*‐test were utilized for the comparison between two groups. One‐way ANOVA with Tukey post‐test were utilized for the comparison among three and more groups. The value of *p* < .05 was recognized statistically significant. *p < .05, **p < .01, and ^#^ *p* < .05.

## 3 RESULTS

### 3.1 NEAT1 and YAF2 were increased, pyroptosis was activated, but miR‐5047 was decreased in a cell model of PD

To investigate expression of NEAT1, miR‐5047, and YAF2 in PD, we established a cell model of PD with SH‐SY5Y cells through MPP^+^ induction. Expression of NEAT1 and YAF2 mRNA were increased, while miR‐5047 was decreased in the SH‐SY5Y cells treated with MPP^+^ (Figure 1A). Western blotting assay results also indicated that YAF2 was increased in the SH‐SY5Y cells treated with MPP^+^ (Figure 1B). Meanwhile, we also detected the activation of NLRP1 inflammasomes‐mediated pyroptosis in MPP^+^‐induced SH‐SY5Y cells. As shown in Figure 1C, cleaved caspase‐1, pro‐caspase‐1, NLRP1 and ASC were highly expressed in the SH‐SY5Y cells treated with MPP^+^. Concentrations of IL‐1β and IL‐18 were higher in supernatant of the MPP^+^‐treated SH‐SY5Y cells than that in the untreated cells (Figure 1D). Overall, expression of NEAT1 and YAF2 was increased, NLRP1 inflammasome‐mediated pyroptosis was activated, while miR‐5047 expression was declined in the SH‐SY5Y cells treated with MPP^+^.

**Figure 1:** Detecting of NEAT1, miR‐5047, YAF2 and pyroptosis‐related proteins. MPP^+^‐treated SH‐SY5Y cells were used to mimic PD in vitro. (A) Expression levels of NEAT1, miR‐5047 and YAF2 mRNA were determined by using qRT‐PCR assay. (B) Expression level of YAF2 protein in MPP^+^‐treated and untreated SH‐SY5Y cells was measured by using Western blot. (C) Expression levels of NLRP1 inflammasomes‐ and pyroptosis‐related proteins including NLRP1, ASC, pro‐caspase‐1 and cleaved caspase‐1 were also analyzed by using Western blot. (D) Concentrations of IL‐1β and IL‐18 in supernatant of SH‐SY5Y cells were analyzed through ELISA assay. Data are presented as mean ± SD of three independent experiments. Student's *t*‐test was used to analyze the significant difference between two independent groups. **p < .01 versus Control group. For these analysis, independent variables are MPP^+^ treatment or no treatment, and dependent variables are the expression level of factors.

### 3.2 NEAT1 increasing aggravated SH‐SY5Y cells pyroptosis induced by MPP^+^

To probe the effect of NEAT1 on the pyroptosis induced by MPP^+^ in SH‐SY5Y cells, we constructed NEAT1 overexpression plasmid and synthetized the specific NEAT1 siRNA. Expression of the NEAT1 was significantly upregulated by transfection of the NEAT1 overexpression plasmid, and was downregulated by transfection of the NEAT1 siRNA (Figure 2A). NEAT1 increasing could enhance cells apoptosis, while NEAT1 decreasing could attenuate cell apoptosis in the SH‐SY5Y cells treated with MPP^+^ (Figure 2B,C). In the SH‐SY5Y cells treated with MPP^+^, NEAT1 increasing facilitated pro‐caspase‐1, NLRP1, ASC and cleaved caspase‐1 expression, but NEAT1 decreasing suppressed expression of above factors (Figure 2D). Consistently, in the SH‐SY5Y cells treated with MPP^+^, NEAT1 increasing promoted secretion of IL‐1β and IL‐18, and NEAT1 silencing reduced secretion of IL‐1β and IL‐18 (Figure 2E,F). In conclusion, NEAT1 promoted pyroptosis in the SH‐SY5Y cells treated with MPP^+^.

**Figure 2:** Exploring of the effects of NEAT1 on MPP^+^‐induced cell pyroptosis. Overexpression of NEAT1 or silencing of NEAT1 in the MPP^+^‐induced SH‐SY5Y cells. Subsequently, (A) expression level of NEAT1 in the cells was measured through qRT‐PCR assay. (B, C) TUNEL staining was carried out to determine the apoptotic rate of SH‐SY5Y cells. Scale bar = 25 μm. Magnification factor is ×40. (D) Expression levels of NLRP1 inflammasomes‐mediated pyroptosis were checked by using Western blot. (E, F) Concentrations of IL‐1β and IL‐18 in supernatant were determined by ELISA assay. Data are presented as mean ± SD of three independent experiments. Statistical significance was tested using one‐way ANOVA with Tukey posttest. **p < .01 versus Control group, ^#^ *p* < .05 versus MPP^+^ group. For these analysis, independent variables are the different treatment to cells, and dependent variables are the expression level of factors or apoptotic rate of cell.

### 3.3 NEAT1 promoted YAF2 expression via inhibiting miR‐5047

Furthermore, our data certificated that NEAT1 increasing declined miR‐5047 level, and NEAT1 decreasing facilitated miR‐5047 expression in the SH‐SY5Y cells treated with MPP^+^ (Figure 3A). NEAT1 increasing boosted YAF2 mRNA and protein expression, and NEAT1 silencing restrained YAF2 mRNA and protein expression in the SH‐SY5Y cells treated with MPP^+^ (Figure 3B,C). Mechanism of competitive endogenous RNAs (ceRNAs) proposes that lncRNAs compete miRNA with mRNA, thus to reduce the inhibition of miRNAs to mRNA.^24^ Here, we predicted the binding sites between NEAT1 and miR‐5047 using starBase v2.0 database (Figure 3D), as well as the binding sites between miR‐5047 and YAF2 3ʹ‐UTR using TargetScan Human database (Figure 3E). Combination of NEAT1 and miR‐5047 was proved by usage luciferase reporter assay (Figure 3F). Combination of miR‐5047 and YAF2 3ʹ‐UTR was also confirmed by luciferase reporter assay (Figure 3G). YAF2 was a downstream target of miR‐5047. To probe whether NEAT1 affects YAF2 expression via miR‐5047, miR‐5047 mimics was co‐transfected with NEAT1 overexpression plasmid into the SH‐SY5Y cells treated with MPP^+^. NEAT1 increasing promoted the YAF2 mRNA expression, which was reversed by miR‐5047 mimics transfection (Figure 3H). NEAT1 increasing‐induced YAF2 protein expression also was partly rescued by miR‐5047 increasing (Figure 3I). In addition, the inhibition of NEAT1 decreasing to YAF2 mRNA and protein expression was reversed by miR‐5047 decreasing (Figure 3J,K). In a word, NEAT1 promoted expression of the YAF2 via sponging miR‐5047.

**Figure 3:** miR‐5047 combined with NEAT1 or YAF2 3ʹ‐UTR. Overexpression of NEAT1 or silencing of NEAT1 in the MPP^+^‐induced SH‐SY5Y cells. Subsequently, (A) expression of miR‐5047 was analyzed by using qRT‐PCR. (B) Expression of YAF2 mRNA was detected by using qRT‐PCR. (C) Western blot was performed to measure expression of YAF2. **p < .01 versus Control group, ^#^ *p* < .05 versus MPP^+^ group. For these analysis, independent variables are the treatment methods of cells, and dependent variables are the expression level of factors. (D) The binding sites between NEAT1 and miR‐5047 was predicted by using starBase v2.0 database. (E) The binding sites between miR‐5047 and YAF2 3ʹ‐UTR was predicted by using TargetScan Human database. (F, G) Combination of miR‐5047 with NEAT1 or YAF2 mRNA was determined through luciferase activity assay. *p < .05. Moreover, NEAT1 overexpression plasmids were cotransfected with miR‐5047 mimics or mimics NC into SH‐SY5Y cells. Then, (H, I) qRT‐PCR and Western blot were performed to determine the expression levels of YAF2 mRNA and protein, respectively. **p < .01 versus Vector group, ^#^ *p* < .05 versus pcDNA‐NEAT1 + mimics NC group. In addition, NEAT1 siRNAs were cotransfected with miR‐5047 inhibitor or inhibitor NC into SH‐SY5Y cells. (J, K) qRT‐PCR and Western blot were performed to determine the expression levels of YAF2 mRNA and protein, respectively. **p < .01 versus si‐NC group, ^#^ *p* < .05 versus si‐NEAT1 + miR‐5047 inhibitor group. Data are presented as mean + SD of 3 independent experiments. Statistical significance was tested using one‐way ANOVA with Tukey post‐test. For these analysis, independent variables are the treatment methods of cells, and dependent variables are the expression level of factors.

### 3.4 Increasing miR‐5047 partly reversed the promotion of NEAT1 to MPP^+^‐induced pyroptosis

Based on above results, we asked that whether NEAT1 enhances the pyroptosis in the SH‐SY5Y cells treated with MPP^+^ through miR‐5047/YAF2 signaling pathway. NEAT1 overexpression plasmid was co‐transfected with miR‐5047 mimics into the SH‐SY5Y cells treated with MPP^+^. Our results certificated that the promotion of NEAT1 to SH‐SY5Y cells apoptosis induced by MPP^+^ was reversed by miR‐5047 increasing (Figure 4A,B). The promotion of NEAT1 to pro‐caspase‐1, NLRP1, ASC, and cleaved caspase‐1 expression also was rescued by miR‐5047 increasing (Figure 4C). In addition, miR‐5047 overexpression rescued the promotion of NEAT1 to IL‐β and IL‐18 secretion in SH‐SY5Y cells (Supporting Information: Figure 1A,B). The promotion of NEAT1 to SH‐SY5Y cells pyroptosis induced by MPP^+^ was rescued by miR‐5047 overexpression.

**Figure 4:** NEAT1 regulates SH‐SY5Y cells pyroptosis through miR‐5047. NEAT1 overexpression plasmids were co‐transfected with miR‐5047 mimics or mimics NC into SH‐SY5Y cells. Subsequently, (A, B) apoptotic rate of SH‐SY5Y cells was detected by using TUNEL staining. Scale bar = 25 μm. Magnification factor is ×40. (C) Expression levels of NLRP1 inflammasomes‐mediated pyroptosis‐related proteins were measured by Western blot. *p < .05 versus MPP^+^ + Vector group, and ^#^ *p* < .05 versus MPP^+^ + pcDNA‐NEAT1 group. Data are presented as mean ± SD of three independent experiments. Statistical significance was tested using one‐way ANOVA with Tukey post‐test. For these analysis, independent variables are the different treatment to cells, and dependent variables are the expression level of factors or apoptotic rate of cell.

### 3.5 YAF2 silencing reversed the promotion of NEAT1 to MPP^+^‐induced pyroptosis

We also co‐transfected the NEAT1 overexpression plasmid with the YAF2 siRNA into the SH‐SY5Y cells treated with MPP^+^. Results indicated that the promotion of NEAT1 to SH‐SY5Y cells apoptosis induced by MPP^+^ was reversed by YAF2 downregulation (Figure 5A,B). Consistently, upregulation of the pro‐caspase‐1, NLRP1, ASC and cleaved caspase‐1 induced by NEAT1 was also suppressed by YAF2 decreasing (Figure 5C). The promotion of NEAT1 to IL‐1β and IL‐18 secretion in MPP^+^‐treated SH‐SY5Y cells also was rescued by YAF2 decreasing (Supporting Information: Figure 2A,B). In short, the promotion of NEAT1 to SH‐SY5Y cells pyroptosis induced by MPP^+^ was rescued by YAF2 decreasing.

**Figure 5:** NEAT1 regulates SH‐SY5Y cells pyroptosis through YAF2. NEAT1 overexpression plasmids were co‐transfected with YAF2 siRNA or siRNA NC into SH‐SY5Y cells. Then, (A, B) apoptotic rate of SH‐SY5Y cells was detected through TUNEL staining. Scale bar = 25 μm. Magnification factor is ×40. (C) Expression levels of NLRP1 inflammasomes‐mediated pyroptosis‐related proteins were measured by Western blot. *p < .05 versus MPP^+^ + Vector group, and ^#^ *p* < .05 versus MPP^+^ + pcDNA‐NEAT1 group. Data are presented as mean ± SD of three independent experiments. Statistical significance was tested using one‐way ANOVA with Tukey post‐test. For these analysis, independent variables are the different treatment to cells, and dependent variables are the expression level of factors or apoptotic rate of cell.

## 4 DISCUSSION

In the present study, our data demonstrated that NEAT1 is highly expressed in the SH‐SY5Y cells treated with MPP^+^, and it aggravated MPP^+^‐induced pyroptosis through promoting YAF2 expression by sponging miR‐5047. Here, we explored the role of NEAT1 in neuron pyroptosis induced by MPP^+^, and the regulatory mechanism of it in the pyroptosis.

A growing body of studies indicated that lncRNAs are a promising target for PD treatment. Yang et al.^25^ reported that lncRNA HOXA‐AS2 is increased in peripheral blood mononuclear cells of the patients with PD, and it maybe participate in the development of PD through regulating microglial‐mediated neuroinflammation via interacting with the polycomb repressive complex 2. Another lncRNA, lincRNA‐p21, could exacerbate microglial‐mediated neuroinflammation and loss of TH^+^ neuron in the PD mouse model induced by MPTP.^26^ MPTP/MPP^+^ is a typical drug, which has been used for the establishment of PD model. Here, our data showed that expression level of lncRNA NEAT1 is increased in the SH‐SY5Y cells treated with MPP^+^. NEAT1 is a well‐studied lncRNA in multiply disorders. It was reported that NEAT1 is involved in a series physiological and pathological processes, including cancer, immune response, neurodegenerative disorders, and viral infection.^27^ The role and action mechanism of NEAT1 in inflammation‐induced neuron apoptosis in PD, however, has not yet been fully clarified.

Neuroinflammation is one of the major cause of TH^+^ neuron loss in PD, it can be induced by inflammasome‐mediated pyroptosis. Inflammasome is a critical mediator of innate immune response to infection. NLRP1, NLRP3, NLRC4, IPAF, and absent in melanoma 2‐associated inflammasomes are the most well‐known inflammasomes.^28^ NLRP1 inflammasome consists of NLRP1, ASC and pro‐caspase‐1. Inflammasomes induces the activation of caspase‐1, and then activated caspase‐1 cleaves gasdermin D and promotes the releasing of IL‐1β and IL‐18.^29^ In the current study, our data revealed that MPP^+^‐induced NLRP1 inflammasome‐mediated pyroptosis was enhanced by NEAT1 overexpression, but attenuated by NEAT1 downregulation. To explore the regulatory mechanism of NEAT1 to neuron pyroptosis, we predicated the binding sites between NEAT1 and miR‐5047. Our results showed that expression level of miR‐5047 was decreased in the SH‐SY5Y cells treated with MPP^+^. Combination of NEAT1 and miR‐5047 was proved by usage luciferase reporter assay. Meanwhile, our data indicated that the promotory effect of NEAT1 on SH‐SY5Y cells pyroptosis is rescued followed by miR‐5047 overexpression.

Transcription factor Yin‐Yang‐1 (YY1) is a crucial regulator for gene expression, and participates in regulation of many disorders including PD.^30^ It was reported that YY1 could regulate neuroinflammation development through suppressor of cytokine signaling 3.^31^ YAF2 was first identified in a yeast two‐hybrid screen for transcriptional factor of YY1, and was proved to be interacted with YY1 in muscle differentiation and development.^32^, ^33^ At present, the functions of YAF2 in PD remain unreported. In the current present, YAF2 was downregulated in the SH‐SY5Y cells treated with MPP^+^, and was a downstream target of miR‐5047. NEAT1 could promote YAF2 expression by acting as miR‐5047 sponge. Importantly, the promotory effect of NEAT1 on SH‐SY5Y cells pyroptosis was partly rescued by YAF2 downregulation. YAF2 maybe mediate the regulatory of NEAT1 to MPP^+^‐induced SH‐SY5Y cells pyroptosis.

In the current study, MPP^+^‐treated SH‐SYY cells were used to mimics PD in vitro. Our data demonstrated that NEAT1 could aggravate MPP^+^‐induced pyroptosis in SH‐SY5Y cells through promoting YAF2 by sponging miR‐5047. We clarified a novel action mechanism of NEAT1 in the pathogenesis of PD, indicating that NEAT1/miR‐5047/YAF2/pyroptosis axis involved in the development of the disease. These data indicated that NEAT1 is a promising molecular target for PD treatment, and the drugs targeting NEAT1/miR‐5047/YAF2 axis maybe a candidate method for PD treatment. Future investigations are needed to verify the conclusion in current study with the animal models applicable to humans. Whether NEAT1 could regulate development of PD through acting as a molecular scaffold or binding with RNA‐binding proteins. In further, more studies need to be done.

## AUTHOR CONTRIBUTIONS

Hong Shen, Hui Song, and Qiang Sun contributed to the conception of the study and helped perform the analysis with constructive discussion. Hong Shen, Hui Song, Songlin Wang, and Daojing Su performed the experiment; contributed significantly to analysis and manuscript preparation; performed the data analyses. Hong Shen and Qiang Sun contributed to write the manuscript.

## CONFLICT OF INTEREST STATEMENT

The authors declare no conflict of interest.

## Supporting information


**Supplementary information**.

**Supplementary information**.

## Data Availability

All data generated and/or analyzed during this study are included in this published article.
